The article "Environmental Accounting System Model Based on Artificial Intelligence Blockchain and Embedded Sensors" was published in 2022. Journal: Comput Intell Neurosci.

# Environmental Accounting System Model Based on Artificial Intelligence Blockchain and Embedded Sensors

**DOI:** 10.1155/2022/3803566

**Published:** 2022-08-03

**Authors:** Wenyu Zhang, Mengpu Zhu

**Affiliations:** ^1^School of Economics and Management, Nanjing University of Science and Technology, Nanjing 210094, Jiangsu, China; ^2^Metropolitan College, Boston University, Boston, MA 02215, USA

## Abstract

With the rapid development of communication technology and automation technology, sensors are becoming more and more intelligent. This study proposes an environmental accounting system model based on artificial intelligence blockchain and embedded sensors. A high-precision sensor system based on embedded technology is first built, which not only avoids the shortcomings of analog data transmission, but also has high performance and price advantages. At the same time, it can be easily combined into a simple sensor network, and array measurement can be realized through the development of blockchain technology. However, the current blockchain system has the disadvantage of storage limitation. The problem is particularly serious when a large amount of data needs to be stored in the blockchain, especially when the blockchain is combined with big data. As a comprehensive field of accounting, ecology, and environmental science, environmental accounting has made great contributions to sustainable development in the field of accounting. The theoretical research in the field of environmental accounting in China started late, and a unified environmental accounting system has not actually been established. Under the conditions of immature theoretical and policy basis, companies have almost no actual surveys on environmental accounting. The characteristics of blockchain technology, such as decentralization, transparency, and changes in information unavailability, can fully solve the problem that the current accounting information system cannot consolidate transaction information and the accounting process. The reliability assurance mechanism of the accounting information system based on blockchain technology can greatly ensure the reliability of the accounting information system, effectively suppress accounting fraud, and improve the transparency of information.

## 1. Introduction

With the development of industry and technology, more and more industrial manufacturing processes need to be smarter and more accurate. In order to optimize the process and production process, in order to provide reliable information, industrial production needs more accurate and smarter sensors to provide indispensable conditions for the development of industrial automation [1]. With the development of intelligence, sensors must break the traditional condition of relying only on analog output to provide a single test [2]. In order to provide omnidirectional real-time sensor output for industrial automation, more and more embedded systems need to be cascaded to form a simple sensor network [3, 4]. This study takes into account the influence of noise and especially considers anti-interference technology in the design of the sensor, so that the output of the sensor has a high antinoise performance [5]. In addition, blockchain technology is also becoming a very valuable frontier technology field through its unique technical advantages, innovative value, intellectual property rights, network finance, medical care, insurance, internet of things, and other wide-ranging applications [6]. It is becoming a very valuable frontier technology field and has a huge influence [6]. As a value transfer protocol, blockchain technology is applicable to all fields related to value. Since the reform and opening up, China's national economy has rapidly developed [7]. However, due to the relatively rapid progress of China's industrialization, the price of rapid development is the destruction of the ecological environment and the excessive consumption of energy. Next, we will face more and more serious environmental pollution and insufficient resources [8]. In the trend of global environmental issues, the external pressure on enterprises to be responsible for environmental protection is increasing, and it is inevitable for society to establish an environmental accounting system in the future. Effective environmental accounting can strengthen the supervision and implementation of environmental departments, promote the rational development and utilization of natural resources, reduce damage to the environment, and achieve the goal of sustainable development. However, the traditional accounting system only pays attention to the economic activity accounting of the enterprise and ignores the accounting content related to the environment. In this context, ecological environmental protection and pollution prevention should also become the main content of the accountant's responsibility [9–12]. Therefore, in the field of accounting, environmental accounting has not formed a systematic study due to its imperfect content, and there are big problems in the application process.

Based on the above background, in order to further deepen the knowledge related to the construction method of environmental accounting system and enrich the theoretical research of environmental accounting, this study proposes an environmental accounting system model based on artificial intelligence blockchain and embedded sensors, constructs a series of environmental accounting systems, and applies them to specific projects.

## 2. Related Work

In the literature, the types of blockchain technologies applicable to the accounting industry are combined with other new technologies to establish an accounting information system that includes a blockchain-based accounting process model [13]. The company's revenue and expenditure accounting is represented, using blockchain technology, to improve accounting identification, improve accounting measurement, research and produce three-entry bookkeeping methods including economic action records, and provide more comprehensive and multidimensional real-time accounting reports based on the basic principles of blockchain, information asymmetry theory, and moral crisis [14]. The literature believes that the current accounting information system cannot guarantee the processing of original transaction information, and the quality is worrying [15].

Facts have shown that 53 listed companies have used the insufficiency of the reliability guarantee mechanism of the accounting information system, and financial frauds have occurred that tampered with transaction facts. Therefore, it proves once again that the current accounting information system is unreliable. Research on the measurement principle of piezoresistive mechanical sensors has been carried out in the literature [16]. The hardware circuit of the high-precision mechanical sensor based on the embedded system is designed in detail from reality. Aiming at the problem of government data sharing, data exchange through blockchain is recorded in the literature. We use aperture, fingerprint, and other authentication methods to authenticate users, and add smart configuration to prevent illegal use. We use virtual currency to promote sharing and increase the enthusiasm for data sharing [17]. Enterprise B is selected as the example enterprise, analyzes the problems existing in the environmental cost calculation of B automobile manufacturing enterprise, and proposes an executable solution. We enter MFCA, and calculate the environmental cost by combining the accounting object and process decision, cost classification, data collection, the calculation of the internal environmental cost in production, and the lime analysis method to measure the external environment [18]. We obtain loss cost and environmental cost accounting results. According to the actual situation of the enterprise, the literature adopts the mode of setting the second-level theme related to the environment on the basis of maintaining the existing accounting of the enterprise. Second, we apply the accounting system to *A*'s main project *W* project and analyze its application effects [19]. Finally, companies must better integrate environmental accounting systems into future accounting. In the literature, the contour matching algorithm of the embedded vision sensor is designed and implemented, characterized according to the shape gradient, and optimized according to the characteristics of the embedded system, with high-speed matching speed, lighting robustness, versatility, configuration possibilities, etc. as advantages [20]. Software programming is composed of graphics, with Ethernet and fieldbus communication interfaces, to simplify the complex vision measurement system into an easy-to-use intelligent vision measurement sensor suitable for industrial applications [21, 22].

## 3. Embedded Sensors and Artificial Intelligence Blockchain

### 3.1. Embedded Sensors

When the wire length is *l*, the cross-sectional area is *s*, the resistivity is *ρ*, and the resistance is as follows:

(1) $$\begin{array}{c} R=\rho \frac{l}{S}. \end{array}$$

To find the partial derivative of the above formula, the following formula is obtained:

(2) $$\begin{array}{c} R=\rho \frac{l}{S}-\rho \frac{l}{S^{2}}S+\frac{l}{S}\rho ,\\ \frac{R}{R}=\frac{l}{l}-\frac{S}{S}+\frac{\rho }{\rho }=\left(1-\frac{S/S}{l/Sl}\right)\frac{l}{l}+\frac{\rho }{\rho }. \end{array}$$

It is deduced as follows:

(3) $$\begin{array}{c} \frac{R}{R}=\left(1+2\mu +\lambda E\right)\varepsilon . \end{array}$$

The sensitivity coefficient of the resistance line is the relative change in the resistance value caused by the unit distortion.

(4) $$\begin{array}{c} K=\frac{\Delta R/R}{\varepsilon }=1+2\mu +\lambda E. \end{array}$$

Among them, within the tensile limit of the resistance wire, it can be proved that the relative change of the resistance is proportional to the distortion.

(5) $$\begin{array}{c} \frac{R}{R}=K\varepsilon . \end{array}$$

The strain gauge composed of the sensitive grid resistance is combined with the elastic body of the test object through a wire connector to form a basic measurement unit. The *K* value used in the production of resistance wires is usually 1.8 to 3.6.

When the sensor does not apply external force, the output of the sensor is as follows:

(6) $$\begin{array}{c} U_{o}=\left(\frac{R_{1}}{R_{1}+R_{2}}-\frac{R_{4}}{R_{3}+R_{4}}\right)U_{E}. \end{array}$$

The change in the bridge output voltage is as follows:

(7) $$\begin{array}{c} U_{o}=\left(\frac{R_{1}+\Delta R_{1}}{R_{1}+\Delta R_{1}+R_{2}-\Delta R_{2}}-\frac{R_{4}-\Delta R_{4}}{R_{3}+\Delta R_{3}+R_{4}-\Delta R_{4}}\right)U_{E}. \end{array}$$

When Δ*R*_1_=Δ*R*_2_=Δ*R*_3_=Δ*R*_4_=ΔR,

(8) $$\begin{array}{c} U_{o}=\left(\frac{\Delta R}{R}\right)U_{E}=\left(\frac{\Delta R}{R}\right)U_{E}=K\varepsilon U_{E}. \end{array}$$

### 3.2. Definition of Artificial Intelligence Blockchain

Blockchain is a new technology system that combines many technologies. Generally speaking, Figure 1 shows the structure of the blockchain system.

In the blockchain system, especially in the cryptocurrency system represented by Bitcoin, the UTXO transaction model is very common. As far as artificial intelligence is concerned, Turing proposed the famous Turing test in 1950. In this test, the human and the machine are separated by asking questions to the machine. For more than 30% of the machine's answers, the machine is considered to have passed the Turing test, which means that the machine possesses human intelligence. Therefore, Turing is called the father of artificial intelligence. The term artificial intelligence was first proposed in 1956. At the same time, early research results emerged, and American universities and the government jointly developed artificial intelligence technology. However, due to the performance limit of computer hardware at that time, the artificial intelligence technology at that time could not solve the problem of practicability, so it received little attention. In the following years, countries have increased their investment in artificial intelligence research, but artificial intelligence technology has not made great progress, and has not experienced the gorge. When the Deep Blue Robot developed by IBM defeated the world chess champion in 1997, artificial intelligence once again attracted people's attention. This activity is called an epoch-making event in the field of artificial intelligence research. Since then, more and more researchers have participated in artificial intelligence research, and the theory, technology, and engineering practice of artificial intelligence have also rapidly developed, and the relationship between artificial intelligence and practical problems has become closer and closer.

From the perspective of the division of research fields, artificial intelligence can be divided into cognitive computing, mechanical learning, and deep learning. Cognitive computing performs correct human brain decision-making through data collection and natural language processing. The main body of machine learning is the research of algorithms, which are related to many fields including probability, statistics, approximation theory, and the theory of algorithm complexity. The core of machine learning is data. We classify a large amount of data, find rules from the data, and continuously improve and optimize. Because the learning algorithm contains many statistical theories, it is also called statistical learning theory.

### 3.3. Algorithm Principle

If the same type of encryption is used, users can directly perform specific algebraic operations on the encrypted text to obtain the result. The same type of password has the following characteristics:

(9) $$\begin{array}{c} E_{pk}\left(m_{1}+m_{2}\right)=E_{pk}\left(m_{1}\right)E_{pk}\left(m_{2}\right),\\ E_{pk}\left(am_{1}\right)=aE_{pk}\left(m_{1}\right). \end{array}$$

In this study, the secret key SK is divided (labeled as SK1, SK2,…, SK*P*) and distributed to the parties, using the *P*(*p*, *t*) threshold Paillier encryption method. If one party correctly decrypts the ciphertext *C*, at least it needs to cooperate with the other party at *t* − 1.

During the decoding process, each partition I (1 ≤ I ≤ *p*) must use the SKI calculation to partially decode *ci* as follows:

(10) $$\begin{array}{c} c_{i}=c^{2{\text{sk}}_{i}},\\ \psi \left(g_{2}\right)=g_{1},\\ G_{1}=g_{1},G_{2}=g_{2}. \end{array}$$

Bilinear is as follows:

(11) $$\begin{array}{c} e\left(u^{a},v^{b}\right)=e{\left(u,v\right)}^{ab}. \end{array}$$

Figure 2 shows the system model. The model component contains data and encrypted data. Data will be encrypted using the Paillier encryption system.

The CA handles important calculations and decentralization, and all parties jointly evaluate the input function, so that the input is not made public. Confidential data are divided into two or more different parts, and neither party can see each other's private data. The CA will decide whether to distribute keys to the user based on the user's credit score.

Credit score users represent credit providers (banks, etc.). In addition to accessing credit rating information, various analysis algorithms (user authentication, etc.) can be executed on data owned by companies and individuals.

Blockchain is a shared public transaction log that the network relies on. By encrypting the data, the hash of the data is stored in the blockchain to prevent information tampering. If some relevant personnel need to save encrypted data together, many participants are needed to check the encrypted data.

This study uses (*p*, *t*) Paillier encryption. The secret key SK is separated (represented as sk1, sk2,…, SK*P*) and divided into *p* parts. When the parties decrypt the ciphertext *C*, at least the other private keys of *t* − 1 need to be aggregated together.

(1) According to
  (12) $$\begin{array}{c} c=E_{pk}\left(m\right)=g^{m}r^{n}\mathrm{mod}n^{2}. \end{array}$$
(2) According to the same type of encryption system, as shown below
  (13) $$\begin{array}{c} E_{pk}\left(m_{1}+m_{2}\right)=E_{pk}\left(m_{1}\right)+E_{pk}\left(m_{2}\right)=g^{m_{1}+m_{2}}{\left(r_{1}r_{2}\right)}^{n}\mathrm{mod}n^{2},\\ E_{pk}\left(am_{1}\right)=E_{pk}{\left(m_{1}\right)}^{a}=g^{am_{1}}r_{1}^{an}m\mathrm{mod}n^{2}. \end{array}$$

Cloud computing is as follows:

(14) $$\begin{array}{c} C=E_{pk}\left(\sum_{k=1}^{K}v_{k}\right)=\prod_{k=1}^{K}E_{pk}\left(v_{k}\right). \end{array}$$

To use the public key *pk* = (*g*, *n*) to encrypt information, we choose a random integer and calculate the ciphertext

(15) $$\begin{array}{c} E_{pk}\left(m,r\right)={\left(N+1\right)}^{m}r^{N}\mathrm{mod}N^{2}. \end{array}$$

We calculate the original information for decryption

(16) $$\begin{array}{c} m=\frac{\left(E_{pk}{\left(m,r\right)}^{\lambda }\mathrm{mod}N^{2}\right)-1}{N}\lambda^{-1}\mathrm{mod}N. \end{array}$$

The scheme given in this study can also use consensus to recover the random number *R* of a given ciphertext.

(17) $$\begin{array}{c} r=c^{N-1\mathrm{mod}\lambda }\mathrm{mod}N,\\ c=E_{pk}\left(m,r\right){\left(N+1\right)}^{-m}\mathrm{mod}N. \end{array}$$

According to the homomorphic nature of the encryption system, we get the following:

(18) $$\begin{array}{c} E_{pk}\left(m_{1},r_{1}\right)E_{pk}\left(m_{2},r_{2}\right)=E_{pk}\left(m_{1}+m_{2},r_{1}r_{2}\right),\\ E_{pk}{\left(m,r\right)}^{k}=E_{pk}\left(km,r^{k}\right). \end{array}$$

The Paillier encryption system is also blind. In other words, you can modify the ciphertext without modifying the corresponding plaintext.

(19) $$\begin{array}{c} E_{pk}\left(m,r_{1}r_{2}\right)=E_{pk}\left(m,r_{1}\right)E_{pk}\left(0,r_{2}\right). \end{array}$$

### 3.4. Performance Evaluation

In Paillier encryption, the public key (*g*, *n*) and the secret key are *λ* = LCM ((*p* − 1), (*q* − 1)), as shown in Figure 3.

Figure 4 shows the time required to encrypt 32-bit data of 64, 128, 256, 512, and 1024 bits with the public key length. As shown in Figure 4, as the key length increases, consumption in the encryption and decryption process gradually increases.

Combining MATLAB and Python, the test results obtained are shown in Figure 5. It can be understood from Figure 5 that in the case of the same multiplication with the same information length, the processing time will be longer if it is obtained under other conditions under the same type of addition. With the confirmation, the length of exponential processing time required for message processing increases, and various formulas for calculating message processing and time difference become larger and larger.

## 4. Research on Environmental Accounting Based on Embedded Sensors and Artificial Intelligence Blockchain

### 4.1. Analysis of Accounting Credibility Guarantee

The questionnaire first analyzes the reliability of the accounting information system from four aspects and the necessity of the guarantee mechanism. After investigating the importance of the corresponding scores of each content, using the questionnaire survey, the scores of each item are added together to obtain the scores of the 4 elements, and the total value is divided by the number of questionnaires sent back. As shown in Table 1, in order to compare the importance levels of the four elements, average scores were obtained for each option category.

Generally speaking, the average score of the four elements is between 4.0 and 4.5, and there is almost no difference in the level of importance. Next, using SPSS software, a description statistics of 15 subitems of specific content was created, as shown in Table 2 for details.

It can be seen from Table 2 that the average value of all items exceeds 4 points, indicating that all subitems are very important. Among them, the quality of accounting information cannot guarantee the authenticity of transaction information; it is easy to be tampered with; transaction information cannot be tracked; and it is more important that the cost of impropriety is very low. Regarding management issues, the supervisory authority cannot fully investigate the credibility of the original accounting information and cannot guarantee that the cost of the supervisory authority is relatively high.

At the same time, SPSS software is used to carry out relevant description statistics, as shown in Table 3 for details.

It can be seen from Table 3 that the average value of all subitems of this project exceeds 4 points. Therefore, each subproject is very important in the application of the biggest advantage of blockchain technology in the accounting information system. However, the most important thing is to consolidate transaction information, ensure the authenticity and reliability of accounting information, and ensure the traceability of transaction records and results. The average score for this subitem is 4.38. Second, the scores of other subprojects are almost the same. Therefore, the characteristics of distributed book blockchain technology, due to the reliability of accounting information and the reliability of protection, guarantee the cost of system trust from a single point of failure and transparent chain technology, according to the characteristics of blockchain technology; unfair costs have become huge; and the possibility of improper accounting has been greatly reduced. The production of transaction information based on traceability requires supervision. The requirements of these four subprojects are very important.

Based on the survey results, further analysis is carried out. This question investigates this question from two aspects, namely, application links and application business modules. Therefore, the survey results on this issue are described and separately counted from two aspects. The detailed results are shown in Tables 4 and 5.

It can be seen from Table 5 that the score value of each subitem of the project exceeds 4 points, and each module is very important for accounting information processing. Through the above analysis, we found that it is very important to build a reliability assurance mechanism for the accounting information system of blockchain technology on a large scale. Therefore, in order to realize this idea, the conditions that need to be met or the difficulties that need to be overcome also need to be further analyzed. Next, based on blockchain technology, we developed a description and statistics on the realization of the reliability assurance mechanism of the accounting information system. The detailed results are shown in Table 6.

### 4.2. Feasibility of Accounting Mechanism

#### 4.2.1. Legal Feasibility

Blockchain technology is under development, and its applications in various fields have not yet been fully developed and not yet matured. Regarding laws and policies, although there is no relevant law yet, the possibility of blockchain technology is highly evaluated by the government and financial regulatory agencies, and it is being considered for use in government services. In recent years, various products based on blockchain technology have appeared one after another. The governments of all countries, including China, are open to blockchain technology. In China's current legal environment, as long as the application of blockchain technology does not harm the public welfare of the society and does not violate laws and regulations, its legitimacy can be guaranteed.

#### 4.2.2. Advantages Brought by Blockchain Technology

1. In order to meet the requirements of data reliability and reliability. Due to the use of blockchain technology, the cost of forgery of each link has significantly increased, and it is almost impossible to achieve forgery.
2. In order to meet the needs and restrictive requirements of the audit and review of relevant agencies, blockchain technology can record the transaction records of each link. After the information is stored through the blockchain, it cannot be changed at a later stage and can be stored for a long time. Inspectors and regulatory agencies can track on-site information to meet work needs. This can solve the traditional audit problem and cannot guarantee the implementation of 100% review of transaction information.
3. The cost of trust is reduced. Due to the application of blockchain technology, all transaction information in the system can be used by all system participants. If the data are incorrect or incomplete, and some of the data may be missing, all participants can see it, thereby reducing the price paid for credit review and reducing the cost of trust.

#### 4.2.3. Application Feasibility

Through the study of the theoretical principles of the blockchain, we can know its action mechanism and working process. Taking into account the advantages and characteristics of the abovementioned blockchain technology itself, it is suitable for accounting information systems, which can completely avoid the improper risks in the current accounting information systems, and greatly improve the reliability and reliability of financial information. By establishing the two-layer blockchain technology of the original transaction link and the accounting information processing link, transaction information can be consolidated from the source and process, and accounting information cannot be changed or tampered with. The above are the related issues. Therefore, by studying the accounting information processing mode, credit mode, the operation principle of blockchain technology, and model design, a reliable accounting information system is established.

### 4.3. Accounting Model

#### 4.3.1. Accounting Confirmation

At present, the accounting basis for the accounting confirmation of enterprises is mainly the accrual system, and some administrative institutions will also adopt the payment realization system. The advantage of the accrual system is that the income and costs of each period are reasonably matched, which makes the profit recognition of each period more accurate. However, the accrual system also has its drawbacks. For example, the artificial distribution of income and costs can be easily manipulated by corporate managers to generate financial fraud (for example, Ruixing Coffee's coupon model inflates sales).

Income and expenses are two important accounting elements in the process of business operation. Profits are calculated through income and expenses, which reflect the business results of the current period. After satisfying certain conditions, the accountant will increase or decrease a certain asset, liability, or equity of the enterprise in accordance with certain standards, such as the income and expenses and expenditures of the enterprise, to complete further accounting and provide accounting for the stakeholders of the enterprise. Since economic business confirmation in the blockchain system is a mechanism for network nodes to jointly verify and confirm, its application in finance can reduce the possibility of managers' manipulating business. At the same time, the traceability and immutability of blockchain technology will make the accounting information of the cash flow statement more reliable and valuable.

A basic sales activity process is shown in Figure 6.

The purchasing department purchases raw materials and puts them into the warehouse; the production department receives raw materials to produce products and puts them into the warehouse; the sales department connects with customers to form a preliminary cooperation intention. After multiple inquiries and quotations, an agreement is reached and a contract is signed; the library management department will transport the finished products out of the warehouse, and the cooperative logistics company will deliver the goods to the customers and obtain the waybill. The finished products are shipped out of the warehouse, and the cooperative logistic company will deliver the goods to the customers and obtain the freight bill; the financial department's invoicing personnel will confirm the income according to the accounting standards and according to the relevant vouchers such as the finished product outbound slips and the outbound slips pushed down by the sales department. We pay the taxes payable and carry forward the relevant costs at the end of the month. If it is sold on credit, it is also needed to confirm the accounts receivable and write off the accounts after receiving the payment.

#### 4.3.2. Accounting Measurement

The current currency measurement of corporate accounting is mainly based on the actual currency issued by the state. In China's accounting law, accounting stipulates that the renminbi is the standard currency for accounting. Income and expenditure are mainly carried out in currencies other than RMB. One of these currencies can be selected as the basic accounting currency, and financial and accounting reports are converted into RMB for calculation. The rapid development of digital currency has affected the original currency measurement model. Central banks of various countries have also begun to study, draft, and implement regulatory measures and laws on digital currencies, and are expected to pilot them, such as the digital renminbi (DC/EP) of the Central Bank of China. As the basic underlying technology of current digital currency, blockchain technology has natural compatibility with digital currency. Therefore, incorporating blockchain technology into the corporate accounting information system and connecting with the blockchain payment and settlement system of the future digital currency can make the company's currency measurement more accurate and efficient, and it is beneficial to the currency cash flow of economic behavior and business and to avoid fraudulent means such as related transactions and self-transactions.

The influence of blockchain technology on currency measurement is also reflected in another aspect. Although currency measurement is currently the most efficient measurement unit, there are still and exposed defects in the development process: factors such as corporate R&D capabilities, human resources, goodwill, intellectual property, and other factors that create corporate value that cannot be accurately measured in currency. Most of the current solutions are supplementary disclosures in the statement notes, but this is not easy for relevant stakeholders to obtain information; another example is that the accounting information of currency measurement is highly specialized, and business departments and their stakeholders may not be able to interpret in an intuitive way the information it needs. Using blockchain technology, the data storage of resource information in various dimensions of economic business in the measurement process will give a wider range of value connotations to the various economic resources and economic activities of the enterprise. For example, the relevant information can be transformed into a functional token such as utility token in the blockchain (the token itself has no intrinsic value; it can only be used as a kind of information; or the price is determined by market supply and demand) and stored in a distributed ledger. The ledger can be traced, and the key query can be used through a certain authorization mechanism, which will help the business and financial personnel to deepen the understanding of corporate accounting information and promote the realization of business and financial integration.

#### 4.3.3. Accounting Records

Looking back at the development of accounting records, bookkeeping has gone from the initial single-entry bookkeeping method to the most widely used double-entry bookkeeping method nowadays, and then to various explorations of the three-entry bookkeeping method. The core purpose of the continuous reform of accounting records can be summarized as follows: two aspects: one is to increase the ability of accounting information to correct errors and avoid accounting fraud, and to improve the authenticity and credibility of accounting information through further development of accounting records; the second is to increase the dimension and breadth of accounting information so that the apparent financial data and business are more closely integrated to improve the relevance of accounting information.

Although Ijiri's three-entry bookkeeping method has created a new idea of considering the driving factors of enterprises to achieve wealth in the book, it lacks inherent rigor, and the mathematical differential relationship between concepts cannot withstand scrutiny. Ijiri confuses the formula to a certain extent. With the concept of dimension, the increase in the “style” of accounting bookkeeping should come from the increase in the “dimensions” of accounting bookkeeping, which can increase the “behavior” that causes changes in assets and equity as a new dimension for the study of three-style bookkeeping. Grigg believes that it is possible to introduce an intermediate agent to perform three-entry bookkeeping through key algorithms and digital signatures.

#### 4.3.4. Accounting Presentation

Accounting presentation is a document that reflects the financial status of an enterprise on a specific date. Due to the limited range of energy of accounting staff, generally based on the basic assumptions of the accounting period, the work of reviewing and closing accounts, sorting out and binding vouchers, etc. are carried out on a regular basis. Accounting reports formed based on this work also come in various forms. The current accounting presentation model has three main problems: first, the report is limited by time and lacks timeliness. The internal and external report users of the enterprise can only understand the accounting information in the report at the time of the previous accounting report and cannot grasp the current time in real time. The second is that the existing accounting presentation model is relatively simple, mainly derived from the static financial data in the traditional double-entry accounting method, and the report user cannot directly generate a clear connection of accounting information and economic and business information Luckin Coffee's 2.2 billion financial fraud incident and its financial report last year were still not disclosed on time at the time of publication of the paper, which not only caused a rapid stock price drop and harmed corporate interests, but also undermined investor confidence and market economic order. The key to the reshaping of accounting presentation by blockchain technology is that it provides technical support for the realization of comprehensive multidimensional and reliable real-time accounting presentation.

## 5. Conclusions

We use cloud storage to expand blockchain storage, and the Paillier cryptographic system to protect the privacy of data shared by multiple parties. If the Paillier cryptosystem is applied to the blockchain, confidential information can be effectively protected and the privacy protection problem of the blockchain can be solved. When operating ciphertext, the Paillier cryptosystem of the same type takes a relatively short time and is more effective. According to the analysis, it is shown that this scheme has high security. Applying blockchain technology to the accounting process, starting from the four processes of economic business confirmation, measurement, recording, and presentation, can enhance the communication between accounting information and economic behavior, and return accounting information to the essence of business. Such an accounting model based on blockchain technology can help financial data to be connected with currency cash flow and the internet of things in real time. It can effectively reduce revenue recognition and expense fraud that may exist in the Luckin Coffee incident. The retrospective monetary cash flow avoids fraudulent means of enterprise-related transactions, thereby promoting the quality of accounting information.

## Figures and Tables

**Figure 1:** Regional chain infrastructure.

**Figure 2:** System model.

**Figure 3:** Paillier key generation time.

**Figure 4:** Paillier encryption and decryption into time.

**Figure 5:** Paillier homomorphic time.

**Figure 6:** Flowchart of corporate sales activities.

**Table 1:** The ranking of the problem categories that restrict the current development of accounting informatization.

Project	Total score	Number of subitems	Total sample size	Mean	Sort
Accounting information quality issues	4300	5	196	4.38	1
Control issues	3336	4	196	4.27	2
Security issues	2484	3	196	4.23	3
Cost issue	2367	3	196	4.02	4

**Table 2:** Descriptive statistics of various subitems.

Specific project	Sample size	Minimum	Max	Mean	Standard deviation
The cost of fraud is very low	196	2	5	4.31	0.755
The original accounting information cannot be fully reviewed	196	1	5	4.30	0.803
The transaction information cannot be traced back	196	2	5	4.17	0.690
The review cost is too high	196	2	5	4.29	0.780
The system is paralyzed by the attack	196	1	5	4.35	0.777
Data center is easily stolen	196	2	5	4.23	0.710

**Table 3:** Descriptive statistics on the level of importance of the greatest benefits brought by the application of blockchain technology in accounting information systems.

Specific project	Sample size	Minimum	Max	Mean	Standard deviation
Increase the cost of fraud	196	1	5	4.25	0.784
Reduce the cost of trust	196	2	5	4.26	0.689
Ensure that the system is not affected by a single point of failure	196	2	5	4.30	0.735

**Table 4:** Descriptive statistics of where blockchain technology should be applied in the accounting information processing process.

Specific project	Sample size	Minimum	Max	Mean	Standard deviation
Original transaction information generation link	196	1	5	4.42	0.777
Accounting information processing link	196	2	5	4.35	0.716
Account book generation link	196	1	5	4.16	0.792
Report generation link	196	1	5	4.217	0.716
Financial information analysis link	196	1	5	4.28	0.785

**Table 5:** Descriptive statistics of which business module should apply blockchain technology in the accounting information processing process.

Specific project	Sample size	Minimum	Max	Mean	Standard deviation
Purchasing module	196	1	5	4.42	0.777
Production module	196	2	5	4.37	0.716
Sales module	196	1	5	4.16	0.794
Other personalized modules customized by theenterprise according to its own needs	196	2	5	4.26	0.726

**Table 6:** Descriptive statistics to realize the concept of the credibility guarantee mechanism of the accounting information system based on blockchain technology.

Specific project	Sample size	Minimum	Max	Mean	Standard deviation
“Internet +” is developing rapidly and is in a fully interconnected environment	196	1	5	4.84	0.773
There is a realistic basis for realizing the idea	196	2	5	4.13	0.682
Regulators need to approve this idea	196	2	5	4.31	0.676

## Data Availability

The dataset can be accessed upon request.
